The article "Ethnomedicinal Use, Phytochemistry, and Other Potential Application of Aquatic and Semiaquatic Medicinal Plants" was published in 2022. Journal: Evid Based Complement Alternat Med.

# Ethnomedicinal Use, Phytochemistry, and Other Potential Application of Aquatic and Semiaquatic Medicinal Plants

**DOI:** 10.1155/2022/4931556

**Published:** 2022-08-10

**Authors:** Ashish Kumar Arya, Medha Durgapal, Arachna Bachheti, Deepti, Kamal Kant Joshi, Yilma H. Gonfa, Rakesh Kumar Bachheti, Azamal Husen

**Affiliations:** ^1^Department of Environment Science, Graphic Era (Deemed to be University), Dehradun, Uttarakhand, India; ^2^Department of Botany and Microbiology, Gurukula Kangri (Deemed to be University), Haridwar, India; ^3^Department of Environmental Science Graphic Era Hill University, Dehradun, Uttarakhand, India; ^4^Department of Industrial Chemistry, College of Applied Science, Addis Ababa Science and Technology University, Addis Ababa, P.O. Box-16417, Ethiopia; ^5^Centre of Excellence in Nanotechnology, Addis Ababa Science and Technology University, Addis Ababa, P.O. Box-16417, Ethiopia; ^6^Wolaita Sodo University, P.O. Box-138, Wolaita, Ethiopia

## Abstract

Medicinal plants have been treating various ailments and diseases since ancient times. Aquatic and semiaquatic medicinal plants play an essential role in human welfare to fulfill their daily needs. They have shown biological, pharmacological, nutraceutical, and commercial applications. This review aims to collect and update all recent information on ethnomedicinal, phytochemistry, pharmacological activities, and nanoparticle synthesis and their uses in aquatic and semiaquatic medicinal plants. Original research papers, review papers, short communications, and book chapters on aquatic and semiaquatic plants have been retrieved from PubMed, Web of Science, Scopus, and Google Scholar. Keywords, ethnomedicinal studies, phytochemistry, pharmacological activities, and nanoparticle synthesis from aquatic and semiaquatic medicinal plants are used for the search. Different aquatic and semiaquatic medicinal plants belonging to the families Acanthaceae, Alismataceae, Amaranthaceae, Apiaceae, Araceae, Asteraceae, Boraginaceae, Ceratophyllaceae, Cyperaceae, Fabaceae, Hydrocharitaceae, Lythraceae, Marsileaceae, Menyanthaceae, Nelumbonaceae, Nymphaeaceae, Onagraceae, Plantaginaceae, Poaceae, Polygonaceae, Pontederiaceae, Primulaceae, Scrophulariaceae, and Zingiberaceae have been studied. They are rich in alkaloids, flavonoids, terpenoids, phenolics, saponins, tannins, dietary fiber, glycosidic derivatives, carbohydrates, and proteins. These phytochemicals have been used for their antimicrobial, antioxidant, hepatoprotective, sedative, anticonvulsant, cytotoxic, antiparasitic, and antidiabetic activities. Besides this, various parts of the plants are used as dietary supplements and green nanoparticle synthesis. These plants are also known for their commercial value and are used as an ingredient in some pharmaceutical industries.

## 1. Introduction

Natural products from medicinal plants are known for their various uses, such as treating infectious diseases, biological applications in the industry as ingredients, food additives, and green synthesis of nanomaterials [1, 2]. About 500,000 plants worldwide have a promising potential for their medical activities [3–6]. Great civilizations such as Mesopotamian, Roman, Greek, Inca, Indus valley, Sindhu, Ghati, and Mohanjordo indicated that humans always preferred to live near plants, streams, lakes, and different types of water bodies to get their foods and shelters. For example, various plant species and their parts have been reported to be used as human and animal diets and sources of medicine [1, 7, 8]. Aquatic and semiaquatic plants are found in all ecological zones; however, most are distributed in subtropical and tropical regions. Aquatic medicinal plants can be divided into two categories based on their habitat. They are aquatic plants and semiaquatic plants. Aquatic plants grow mainly in water bodies or floating on water bodies like algae, whereas semiaquatic plants/amphibian plants prefer to grow in submerged water bodies. Aquatic plants can be classified into two categories based on their ethnomedicinal applications and physicochemical effects. Major aquatic medicinal plants have very high medicinal and economic values and are readily available for commercial purposes for different human welfare. Minor aquatic plants are those plants that still contain therapeutic qualities against multiple diseases and disorders, but either lack availability or have little knowledge regarding their pharmacological properties. This is due to the lack of availability of these plant materials, regional applications of plants, and the economic value of plants, unnoticed or overlooked or neglected by the researchers. However, these plants are highly rich in diversified secondary metabolites due to their association with water bodies and weather conditions [9]. Medicinal plants from the wetland ecosystems have played a vital role in the development of the world since the beginning of human civilization [10]. Aquatic and semiaquatic plants have also been reported with significant prospects for commercial and environmental protection by exploring their hidden riches of medicinal properties [11]. These plants are highly diversified in structural adaptations, distribution, and phytochemical compound syntheses, enabling them to thrive in the diet and numerous applications [12] (Table 1). Aquatic and semiaquatic medicinal plants have multifunctional bioactive compounds widely used to protect against human and livestock health disorders [41].

Aquatic and semiaquatic medicinal plants and their phytochemicals have been widely practiced as traditional medicines worldwide. For instance, 50–60% of people in India live closer to aquatic bodies and use these plants for various practices such as medicinal, ornamental, and religious offspring [10, 41]. Recently, the research interest in aquatic and semiaquatic plants has grown tremendously, increasing the screening of new possible phytoconstituents and the usage of bioactive compounds in approved pharmaceutical drugs. Various literature reports also demonstrated that plants possess high nutritional values, medicinal uses, and several biological and pharmacological activities due to their production of potentially bioactive compounds [46]. Despite the wide range of published documents on aquatic and semiaquatic medicinal plants, the information is scattered and unavailable in one place. Therefore, this review aims to bring all the published documents in one place in the form of a review paper.

## 2. Some Significant Aquatic and Semiaquatic Medicinal Plants

### 2.1. *Acorus calamus (Sweet Flag)*

Sweet flag is an important aquatic medicinal plant belonging to the Araceae family, as shown in Figure 1. It is distributed in marshy areas, shallow lands, and ponds of tropical and subtropical areas such as Asia, Europe, and America [47, 48]. This herb has been used in the Indian Ayurvedic medical systems from earlier civilizations. Many parts of this plant, such as rhizomes, roots, and leaves, are used for their medicinal properties. Sweet flag has been used to treat skin disorders, epilepsy, asthma, diarrhea, hysteria, insanity, insomnia, melancholia, neurasthenia, heart disease, and lung cancer [10]. It contains medicinally essential alkaloids such as choline, acorin, calamine A, bitter glycosides, caramel, gum, resin, and starch tannins [47, 49]. The primary chemical constituents such as *β*-asarone (27.4–45.5%), acorenone (20.86%), and isocalamendiol (12.75%) are reported from its leaves and rhizomes, respectively [50, 51].

### 2.2. *Ageratum conyzoides (White Weed)*

This semiaquatic plant species belong to the Asteraceae family (Figure 2), distributed in tropical and subtropical regions, including Brazil [52]. It is common in Asia, West Africa, and South America. Its leaves and shoots treat fresh cuts and injuries and are used in preparing traditional hair lotion. It also treats pneumonia, wound healing, and skin diseases. Some secondary metabolites also found in the plant are rutin, quercitrin, avicularin hyproside, and catechin [53].

### 2.3. *Ammannia baccifera (Monarch Redstem)*

This semiaquatic medicinal plant belongs to the Lythraceae family (Figure 2), distributed commonly throughout India [54]. The plant treats fever, hepatoprotective activities, rheumatic pains, ringworm, scabies, skin diseases, skin itching, and typhoid fever and possesses antioxidant, larvicidal, and antisteroidogenic properties [55]. The plant has secondary metabolites such as 4-hydroxy-*α*-tetralone, tetralin-4O-*β*-D-glucopyranoside, and ammaniol [56].

### 2.4. *Amomum aromaticum (Namra)*

This aquatic medicinal plant belongs to the Zingiberaceae family (Figure 1), distributed in Bhutan, North East India, and Nepal [57]. It is a common spice and food flavoring agent in Vietnam and other Asian countries [58]. Seeds of the plant exhibit medicinal value for controlling blood pressure. The stem of this plant is consumed in a vegetable diet in Manipur [57]. The plant contains secondary metabolites such as 1,8-cineole, *β*-myrcene, *α*-terpineol, terpinene-4-ol, *α*-pinene, and *β*-pinene [59].

### 2.5. *Bacopa monnieri (Water Hyssop)*

This aquatic plant species belong to the Plantaginaceae family and is native to India, the United States, East Asia, and Australia, as shown in Figure 1. This aquatic plant's leaves and flowers treat asthma, bronchitis, Alzheimer's disease, hypoglycemia, leprosy, ringworms, stomach diseases, blood pressure, and anxiety [60]. The plant contains secondary metabolites, including bacopa saponins such as bacopasaponin F, bacopasaponin E, bacopaside III, bacopaside IV, bacopaside N1, and bacopaside V. Additionally, the plant species has been reported to contain phytoconstituents like monnierin, brahmin, herpestine, *β*-sitosterol, betulinic acid, luteolin, apigenin, D-mannitol, hersaponin, and stigmasterol [61].

### 2.6. *Centella asiatica (Indian Pennywort)*

This aquatic medicinal plant belongs to the Apiaceae family (Figure 1), found in most tropical and subtropical countries, including India, Pakistan, Sri Lanka, Madagascar, South Africa, South Pacific, and Eastern Europe [62]. Leaves, flowers, and fruits of the plant have many medicinal uses and are used to treat various skin diseases, fever, strangury, and brain health [63–65]. The active phytoconstituents found in this plant include triterpenes hydrocarbons [66].

### 2.7. *Centipeda minima (Spreading Sneezeweed)*

This aquatic medicinal plant belongs to the Asteraceae family (Figure 1). It is found in wet places and the rice fields of most Asian countries [67]. The leaves and roots of the plant are used to treat various diseases. It is widely used for antibacterial, antioxidant, anti-angiogenic, and anticancer activities [68, 69]. It contains secondary metabolites such as lactones, sesquiterpenes, and triterpenes [70].

### 2.8. *Ceratophyllum demersum (Coontail)*

This semiaquatic medicinal plant belongs to the *Ceratophyllaceae* family (Figure 2). The plant is found in ponds, ditches, lakes, and quiet streams. Leaves treat diarrhea, fever, dysentery, ulcer, wounds, burning sensation, hemorrhoids, piles, intrinsic hemorrhages, epistaxis, hyperdipsia, and haematemesis. It also cures scorpion stings and bile secretion [18]. The plant contains various secondary metabolites such as alkaloids, cardiac glycosides, tannins, and flavonoids [71].

### 2.9. *Coix lacryma-jobi (Job's Tears)*

This aquatic medicinal plant belongs to the Poaceae family (Figure 1). It is distributed throughout Asian countries and is a native plant of Southeast Asia. Leaves, flowers, and fruits are used as a diet supplement to treat chicken pox, stomachache, and menstrual disorders [33]. It is also reported to possess analgesic and antispasmodic properties [72]. The plant contains triglyceride, *β*-sitosterol, stigmasterol, and phytyl fatty acid ester [73].

### 2.10. *Eclipta prostrate (False Daisy)*

This semiaquatic plant belongs to the family of Asteraceae (Figure 2). It is a native plant of Asia and is also distributed in tropical, subtropical, and warm temperate regions of the world [74]. The plant is used to cure eczema, headache, jaundice, mental disorders, scorpion sting, skin diseases, snakebite, spleen enlargements, and toothache. It also showed antiulcer properties. Secondary metabolites present in this plant are triterpenoids, thiophenes, coumestans, flavonoids, and steroids [75].

### 2.11. *Eleocharis dulcis (Water Chestnut)*

This semiaquatic medicinal plant is commonly known as the Chinese water chestnut and belongs to the Cyperaceae family (Figure 2). The plant is commonly grown as a vegetable in Japan, China, India, and other Asian countries [76]. The plant contains phytochemicals such as carbohydrates, flavonoids, proteins, and minerals [77]. The plant treats amenorrhoea, hernia, nausea, abdominal pain, cardiac risks, liver problems, constipation, pharyngitis, laryngitis, hypertension, and chronic nephritis [74, 78].

### 2.12. *Enhydra fluctuans (Water Cress)*

This aquatic medicinal plant belongs to the Asteraceae family (Figure 1). The plant grows in the marshy areas of tropical and subtropical regions of Asia and Africa [79]. This plant species prefers to grow along with ponds, waterways, ditches, and rice fields [80]. Leaves of the plant are a rich source of protein and are used to treat diseases such as nervous diseases [81], skin diseases, and smallpox [82]. The plant leaves possess antioxidant properties [83]. The plant consists of various secondary metabolites: ethyl acetate, n-butanol, baicalein-7-O-glucoside, and baicalein 7-O-diglucoside [84].

### 2.13. *Hedychium coronarium (White Ginger Lily)*

This aquatic medicinal plant belongs to the Zingiberaceae family (Figure 1). It is a medicinal plant of tropics and subtropics that grows closer to the rivers, streams, or shallow water systems [53]. The plant consists of active constituents such as *β*-transocimenone, linalool, 1,8-cineole, *α*-terpineol, 10-epi-*γ*-eudesmol, sabinene, terpinene-4-ol, 2,8-diene, and *γ*-terpinene [85]. Leaves and flowers have a high potential for fatty acids and are used to treat hair, skin, headache, lancinating pain, inflammatory, intense pain, cough, fever, and cancer [15, 86].

### 2.14. *Heliotropium indicum (Indian Heliotrope)*

This semiaquatic medicinal plant belongs to the Boraginaceae family (Figure 2). The plant is known as Indian heliotrope, distributed in tropical, subtropical, and warm temperate zones [87]. Flowers, shoots, and whole plant parts exhibit medicinal properties and treat asthma, boils, bronchitis, cataract, dysentery, menstrual blood loss, redness and conjunctivitis of the eyes, antiseptic, scorpion sting, and ulcers [88]. The plant possesses phytochemicals such as alkaloids, carbohydrates, proteins, flavonoids, phenolics, glycosidic derivatives, saponins, and phytosterols [89].

### 2.15. *Hydrocotyle sibthorpioides (Lei/Lai-Peruk)*

This aquatic medicinal plant belongs to the Apiaceae family (Figure 1). It is distributed in Southeast Asia and shows various adaptations in different habitats, from terrestrial land to submerging underwater [10]. Leaves of this plant have medicinal values; the juice of fresh leaves is used to treat cough, fever, jaundice, and throat pain [90, 91]. The plant species contains some secondary metabolites such as methyl-ester-3-nitro-propanoic acid, 5-ethyl-4-methyl-5-hepten-3-one, 1-cyclohexyl-2-methyl-2-propanol, and 2-methyl-5-(1-adamantyl) pentan-2-ol [92].

### 2.16. *Hygrophila schulli (Marsh Barbel)*

This semiaquatic medicinal plant belongs to the Acanthaceae family (Figure 2), distributed in Sri Lanka, Myanmar, Indonesia, Malaysia, and the plains of India [93]. Leaves, roots, seeds, and whole plants have many medicinal values. They treat anemia, blood pressure, kidney stone, jaundice, gout, hepatic obstruction, impotence, inflammation, pain, rheumatism, spermatorrhoea, and urinary infections. The secondary metabolites present in the plant arequercetin, apigenin-7-oglucuronide, apigenin-7-O-glucoside, luteolin, luteolin-7-O-rutinosides, and gallic acid [94, 95].

### 2.17. *Limnophila aromatica (Rice Paddy Herb)*

This semiaquatic medicinal plant is known as the rice paddy herb and belongs to the family Plantaginaceae, as shown in Figure 2. It is widely used in Southeast Asia, including Vietnam, Malaysia, and Thailand [96]. It treats various diseases such as dysentery, elephantiasis, fever, indigestion, intestinal worms, menstrual problems, and mucus removal. The plant also has antimutagenic and antitumor properties. It contains starch, dietary fiber, protein, polysaccharides, and lignin [97].

### 2.18. *Ludwigia adscendens (Water Primrose)*

This semiaquatic medicinal plant belongs to the *Onagraceae* family (Figure 2). The plant species cure dysentery, skin diseases, and ulcers. The whole plant has been reported for its emetic, laxative, anthelmintic, antidysenteric, anti-inflammatory, antioxidant, and antimicrobial properties [82]. Phytochemicals such as squalene, betulonic acid, betulin, betulinic acid, and quercetin derivatives are some constituents reported from the plant extract [98].

### 2.19. *Marsilea minuta (Water Clover)*

This aquatic medicinal plant belongs to the Marsileaceae family (Figure 1). It is popularly known as water clover and is distributed worldwide [99, 100]. Leaves of the plant are used to treat headaches, migraine, respiratory diseases, hypertension, muscle tension, and sleeping disorders [101–103]. They also treat chronic cancer and cardiovascular diseases [104]. The leaves and roots of this plant have medicinal values to treat indigestion, kidney infection, nose bleeding, diarrhoeal, cough, hepatitis, headache, hypertension, insomnia, sleeping disorder, and skin diseases [105]. The plant species is also known for its potent antioxidant and antibacterial activity [106]. It consists of many secondary metabolites such as carotenoids, flavonoids, cinnamic acids, benzoic acids, folic acids, ascorbic acids, tocopherols, and tocotrienols [107, 108].

### 2.20. *Nelumbo nucifera (Indian Lotus)*

This aquatic medicinal plant belongs to the Nelumbonaceae family (Figure 1). The plant species are cultivated due to their high commercial value for their medicinal property [109] and as ornamental plants in China, Korea, Japan, India, and Australia [110]. Stems and leaves of the plant have high medicinal values. They are used for the treatment of many diseases such as cough, hypertension [111], urinary problems [13, 41], blood vomiting, piles, and eye vision [15]. Secondary metabolites found in the plant include kaempferol-3-robinobioside, quercetin-3-neohesperidose, nelumborines A, higenamine, quercetin-3-O-glucuronide, syringetin-3-O-glucoside, and 4′-O-*β*-d-glucoside [112].

### 2.21. *Nymphaea nouchali (Blue Water-Lily)*

This aquatic medicinal plant belongs to the Nymphaeaceae family, as shown in Figure 1. Plant parts such as leaves, roots, rhizomes, fruits, flowers, and tubers treat liver, kidney, and heart diseases. It is also known for antimicrobial, antidiabetic, and antioxidant activities [113, 114]. It is widely distributed in South Asian countries, Australia, and Africa [115]. Plant extracts are reported to contain rutin, catechin, myricetin, ellagic acid, gallic acid, vanillic acid, rosmarinic acid, p-coumaric acid, quercetin, and ascorbic acid [116, 117].

### 2.22. *Nymphaea pubescens (Pink Water-Lily)*

This semiaquatic plant belongs to the Nymphaeaceae family (Figure 2). The plant species are distributed in tropical and temperate regions [118]. Rhizome and plant roots cure many diseases and ailments such as abortion, blood dysentery, dyspepsia, jaundice, blood purifier, cystitis, nephritis, fever, insomnia, hemorrhoids, leucorrhoea, menorrhagia, and piles [119]. It contains secondary metabolites such as flavonoid and phenolic compounds [120].

### 2.23. *Persicaria hydropiper (Water Pepper)*

This aquatic medicinal plant belongs to the Polygonaceae family (Figure 1). It shows wide distribution worldwide [121] and grows in marshes, wet areas, and agricultural fields [122]. Leaves and roots of the plant species are used to cure many diseases such as uterine disorders [123], menstrual irregularities, and headaches. The plant contains various secondary metabolites such as (+)-catechin, (−)-epicatechin, hyperin, isoquercitrin, kaempferol, quercetin, rhamnazin, rutin, sesquiterpenes, 3-*β*-angeloyloxy-7-epifutronolide, apigenin-7-O-glucoside, galloyl kaempferol-3-O-glucoside, *α*-pinene, *β*-pinene, 1,4-cineol, fenchone, *α*-humulene, *β*-caryophyllene, and trans-*β*-bergamotene [121].

### 2.24. *Pistia stratiotes (Water Lettuce)*

This aquatic medicinal plant belongs to the Araceae family (Figure 1). The plant species are commonly found in stagnant water (lakes and rivers) throughout Asia and subtropical Asia, Africa, and America [124]. The leaves and roots of the plant have very high medicinal values and are used for curing many diseases such as kidney disorders, leprosy, dysentery, eczema, and ulcers. Its extracts contain secondary metabolites such as phenolics and tannins [125].

### 2.25. *Rotula aquatic (Aquatic Rotala)*

This aquatic medicinal plant belongs to the Boraginaceae family (Figure 1). The plant species is native to India, China, and Malaysia and is also found in Africa and South America [126]. The plant species is a remedy for blood disorders, coughs, dysuria, fever, and heart diseases. The plant's leaves and flowers can be used to treat diabetes, bladder and kidney stones, piles, and venereal diseases. [41]. The plant extracts contain secondary metabolites such as allantoin, baurenol, and kaempferol [126].

### 2.26. *Rotala rotundifolia (Roundleaf Tooth Cup)*

This semiaquatic medicinal plant belongs to the Lythraceae family, Figure 2. The plant species are found in South and Southeast Asia, Japan, Africa, Australia, China, India, and North America [127]. The plant extracts are used as antipyretic and antiswelling. The plant species are also used in treating cold, fever, cough, detoxication, diuresis, gonorrhea, menstrual cramps, piles, production in HepA2 cells, and suppression of HBV surface antigen (HBsAg) [43]. The secondary metabolites reported from some extracts of the plant are quercetin 3-O-*β*-D-2″-acetylglucuronide methyl-ester, kaempferol, quercetin, quercetin 3-O-*β*-D-glucuronide methyl-ester, quercetin 3-O-*β*-D-glucuronide, and apigenin [44].

### 2.27. *Rumex maritimus (Torong-Khongchak)*

This aquatic medicinal plant belongs to the Polygonaceae family (Figure 1). It is widely distributed throughout Bangladesh, India, North Africa, and America [128]. The leaves, roots, and stems of the plant have medicinal values. Leaves paste of the plant is applied to cure leucoderma, burns, and injuries [15], and the roots are used to treat diarrhea [128]. 2-Methoxystypandrone is the commonly reported secondary metabolite present in the plant [129].

### 2.28. *Sagittaria sagittifolia (Koukha)*

This aquatic medicinal plant belongs to the Alismataceae family (Figure 1). It is the only native species of the genus *Sagittaria* in Czechoslovakia. The remaining species of this genus occur mainly in tropical and subtropical regions. It predominates in North America, Europe, and Asia [130]. It is mainly found in Asian countries, including China, Bangladesh, Indonesia, Malaysia, Nepal, Sri Lanka, Philippines, Thailand, Vietnam, Cambodia, and India. Root past showed medicinal uses to treat cough and fever. The plant species contain polysaccharides as the main phytochemical components [131].

### 2.29. *Sphaeranthus indicus (East Indian Globe Thistle)*

This aquatic medicinal plant belongs to the Asteraceae family (Figure 1). The plant is widely distributed in India, Sri Lanka, and other continents like Australia and Africa [132]. It prefers to grow in dry or wet places. Various parts of this plant, including seeds, leaves, flowers, and roots, have many medicinal properties widely used to treat disorders like asthma, chest pains, chronic skin diseases, cough, and mental disorders [41]. Triterpenoids, resin, saponins, tannins, and steroids are the primary reported secondary metabolites present in the plant species [133].

### 2.30. *Spilanthes calva (Toothache Plant)*

This semiaquatic plant species belong to the Asteraceae family (Figure 2). The plant species are distributed in some parts of India [134]. Flower head, roots, and whole plant part have medicinal values that cure dysentery, psoriasis, purgative, rheumatism, scabies, stammering in children, tongue paralysis, and toothache. The plant extracts have antioxidant and cytotoxic properties [135]. Saturated and unsaturated alkyl ketones, alkamides, hydrocarbons, acetylenes, lactones, alkaloids, terpenoids, flavonoids, and coumarins are the main phytochemicals present in the extract of the plant species [136].

### 2.31. *Vetiveria zizanoides (Vetivergrass)*

This semiaquatic medicinal plant belongs to the *Poaceae* family (Figure 2). This plant species is cultivated globally in tropical and subtropical regions [137]. The roots and rhizomes of the plant have medicinal properties. They treat burns, colic, obstinate vomiting, diaphoretic, epilepsy, febrifuge, fever, flatulence, headache, mouth ulcer, refrigerant, rheumatism, scorpion sting, and snakebite. [45]. The plant extracts have been reported to possess various secondary metabolites such as *β*-vetispirene, vetiselinenol, khusimol, *β*-vetinene, and *α*-vetivone [138].

### 2.32. Phytochemistry of Aquatic and Semiaquatic Plants

Aquatic and semiaquatic plants contain many phytochemical compounds responsible for their multifunctional properties [139]. Due to their wide-spectrum chemical properties, these plants possess potential medicinal, biological, pharmacological, and other applications [16, 140]. Phytochemical studies on some aquatic and semiaquatic plants revealed various organic compounds with various chemical structures and functional groups. Some phytochemical compounds reported from the extracts of aquatic and semiaquatic plants are given in Figure 3.

## 3. Uses of Aquatic and Semiaquatic Medicinal Plants

Natural products produced by aquatic and semiaquatic medicinal plants are known for their potential biological applications and diet supplements. Aquatic and semiaquatic plants are often used as medicines for many health disorders and diet supplements due to their nutritional values and medicinal uses, and in pharmaceutical industries for producing herbal-based cosmetic products [10]. These plants diversified chemical and biological properties make them medicinally valuable and increase their demand globally. Some previous studies regarding the importance of aquatic and semiaquatic medicinal plants for biological, industrial, and other applications are discussed and presented in Figure 4.

### 3.1. Antimicrobial Activity

Phytochemicals of aquatic and semiaquatic medicinal plants have been reported to possess many antimicrobial properties. The chemical constituents of essential oil from rhizomes of *Hedychium coronarium* have shown a potential antimicrobial activity [85]. *Nymphaea nouchali* flowers effectively against bacteria strains like *Pseudomonas aeruginosa*, *Bacillus cereus*, and *Staphylococcus aureus* [16]. The extracts of *Pistia stratiotes* also displayed a wide range of antibacterial activity against *Escherichia coli* and *Staphylococcus aureus* [141]. The organic solvent extracts of *Sphaeranthus indicus* showed significant antimicrobial activity [142]. The leaves, rootstock, seeds, and stems of *Polygonum glabrum* possess antimicrobial activity [10]. Secondary metabolites from extracts of aquatic and semiaquatic medicinal plants such as *Acorus calamus*, *Centella asiatica*, *Heliotropium indicum*, *Marsilea minuta*, *Sphaeranthus indicus*, *Andrographis peniculata*, and *Clerodendrum viscosum* have been reported by different scholars for their promising antimicrobial activities [60, 64, 85, 88, 106, 142–146].

### 3.2. Antioxidant Activity

Aquatic and semiaquatic medicinal plants are known for their potential antioxidant properties. Earlier reports showed that the reducing power of essential oil of *Hedychium coronarium* might be strongly correlated with their antioxidative activities [85]. Some literature reported that the phytoconstituents of *Bacopa monnieri* showed good antioxidant properties [147]. Epifano and his coworkers (2015) reported that *the Nymphaea nouchali* is a rich source of antioxidants. Potential antioxidant compounds are identified from the extracts of *Centella asiatica*, *Ipomea aquatic, Nelumbo nucifera, Nasturtium officinale, and Ludwigia adscendens*. Phytochemical compounds with antioxidant properties were found in aquatic and semiaquatic plant species such as *Persicaria hydropiper, Rotula aquatic, Sphaeranthus indicus, Polygonum glabrum, Ammannia baccifera, Ipomea aquatic, Nymphaea nouchali, Acorus calamus, Hedychium coronarium, Heliotropium indicum, Marsilea minuta,* and *Vetiveria zizanioides* [107, 148–151].

### 3.3. Hepatoprotective Activity

*Sphaeranthus amaranthoides* methanolic extracts demonstrated significantly higher hepatoprotective activity than control groups [152]. The ethyl acetate extract of *Enhydra fluctuations* was found to have more potent hepatoprotective effects due to its potential flavonoid compounds. Phytoconstituents from *Marsilea minuta* plant species displayed significant hepatoprotective effects [108]. The protective effect of a methanolic extract of *S. indicus* against CCl_4_-induced hepatotoxicity was reported [153]. The ethanolic extract of *Nymphoides hydrophylla* was checked against CCl_4_-induced liver injury in albino rats and demonstrated impressive hepatoprotective activity [154]. Hepatoprotective studies of extracts of *Hygrophila auriculata* checked against HepG2 cells and paracetamol-induced hepatotoxicity and found that it improved hepatoprotective effects. [94]. The ethanolic extract of *Ipomoea aquatic* has been reported to effectively prevent thioacetamide-induced hepatic damage in animal models [155].

### 3.4. Sedative Activity

The natural products from *Marsilea minuta* [108], rhizome extract of *Acorus calamus* [149], and petroleum-ether extract of root parts of *Hygrophila schulli* [95] showed promising sedative activity. *Bacopa monnieri* and *Enhydra fluctuans* plant species have potential sedative actions [156, 157]. The alcoholic extract of *Sphaeranthus indicus* has been reported with significant sedative activity compared to standard sedative pentobarbitone and diazepam in the Swiss albino rat model [142, 153]. In the Ayurvedic system, *the Acorus calamus* plant is known as a magic root due to its sedative effect [158]. Various literature findings displayed that *Cyperus tegetum* has been used by tribal people for the treatment of mental disorders such as epilepsy [159, 160].

### 3.5. Anticonvulsant Activity

Sharma and coworkers (2020) displayed that extracts and compounds from the *Acorus calamus* demonstrated anticonvulsant activity with significant signaling pathways. For instance, methanolic and acetone extracts of *Acorus calamus* leaves have shown promising anticonvulsant activity [161]. The roots and rhizomes of *the Acorus calamus* also possess significant anticonvulsant activity [158]. Several pieces of the literature indicated that *Cyperus tegetum* plant has anticonvulsant activity [159, 160]. The aqueous and alcoholic extracts of roots and rhizomes of *Nymphoide indica* exhibited effective anticonvulsant activity [154]. Hydroalcoholic extract of *Sphaeranthus indicus* plant species showed anticonvulsant effects in the earlier studies [142].

### 3.6. Cytotoxic Activity

Samanta and coworkers (2020) reported that extract from the aerial part of *Ipomea aquatic* showed a cytoprotective role in the liver and other organs [162]. Methanolic and aqueous extracts of the *Acorus calamus* have been known for their cytotoxicity effects [158, 163]. The methanol extract of *Mollugo cerviana, Trichosanthes cucumerina,* and *Vetiveria zizanioides* plants have been reported for their cytotoxicity against cancer cells such as HeLa and MCF-7 cell lines [151]. Alcoholic extracts of *Enhydra fluctuations, Andrographis peniculata,* and *Clerodendrum viscosum* exhibited potent cytotoxicity against brine shrimp compared to ampicillin trihydrate as a positive control [164, 165]. The ethanolic extract of *Centella asiatica* exhibited weak cytotoxicity effects compared to the standard drugs [64].

### 3.7. Antiparasitic Activity

Several studies on aquatic and semiaquatic medicinal plants show their antiparasitic properties. Nymphoides plant species possess antiprotozoal, antimalarial, and anthelmintic properties [154]. Organic solvent extracts of various parts of the genus *Spilanthes*, such as dichloromethane extract of flowers, methanol extract of flowers, and cold dichloromethane extract of plant stems, have been shown to have significant activity against malaria and sleeping sickness diseases [136].

### 3.8. Antidiabetic Activity

Different plant extracts treat diabetes mellitus [166–168]. *Centella asiatica, Hedychium coronarium, Ipomea aquatic*, *Pistia stratiotes, Spergularia marina,* and *Nymphaea nouchali* have been reported as medicinal plants with effective antidiabetic properties due to their potency in the wide range of bioactive compounds [41, 169]. Ethyl acetate extracts and pure compounds obtained from *Acorus calamus* plant species have been reported for their strong antidiabetic effects [170]. The shoots and roots of *Ipomea aquatic* are also used to treat diabetes [171].

### 3.9. As a Dietary Supplement

Several aquatic and semiaquatic plant species are available as food using their various parts, such as stems, leaves, roots, rhizomes, flowers, flower heads, and fruits. For example, the edible part of *Oryza sativa* (rice) is its grain. In contrast, the leaves of *Nasturtium officinale* (Watercress), *Neptunia oleracea* (Water mimosa), and *Oenanthe javanica* (Japanese parsley) are used as human food [117]. Some previous studies revealed that *Enhydra fluctuation*, an edible semiaquatic herbaceous vegetable, is a rich source of phytochemicals such as *β*-carotene and ascorbic acid, which are required in diet supplements [172]. *Ipomea aquatic* is commonly used as a leafy vegetable or salad, which contains medicinally important flavonoids, alkaloids, and carotenes [10]. The leaves, roots, fruits, flowers, rhizomes, and tubers of *Nymphaea nouchali* plant species have been eaten in times of food scarcity [10, 41]. *Ludwigia adscendens* plant has been known to be consumed in the vegetable diet in China [173]. Leaves and tender shoots of the underutilized *Alternanthera sessilis* plant species are used in the vegetable diet for their potential nutritional and medicinal values [174]. Chia and coworkers (2015) reported that the leaves of *the Alternanthera sessilis* plant had been consumed raw or cooked as a food supplement [173]. Seaweeds are used for making a variety of foods. For instance, major aquatic and semiaquatic plant species that have been reported as human food includes *Acorus calamus*, *Aeschynomene aspera*, *Alternanthera philoxeroides*, *Centella asiatica*, *Colocasia esculent*, *Cyperus rotundus*, *Eleocharis dulcis*, *Hydrolea zeylanica, Hygroryza aristata*, *Nymphoides hydrophylla*, *Oryza sativa*, *Pistia stratiotes*, *Polygonum plebeium*, *Trapa natans*, *Vallisneria spiralis*, and *Spilanthes calva* [41].

### 3.10. As Industrial/Commercial Products

The use of macro-algae in pharmaceutical industries showed their importance for humans as they were applied as antibiotic, antifouling, antiviral, anti-inflammatory, cytotoxic, and antimitotic agents. The flour of fruits of *Trapa bispinosa* is reported to have important commercial uses in the milk industry and as a filler in the pharmaceutical industry [169]. Similarly, the rhizome extract and essential oils of the *Acorus calamus* are widely used in the flavoring industry and for commercial purposes [149, 175].

### 3.11. In the Green Synthesis of Metallic Nanoparticles

Nanoparticles have more advanced properties than bulk materials due to their superior behavior with defined shape and size [176]. The increased surface-to-volume ratio and quantum size effect properties of metal/metal oxide nanoparticles are the main reason for their chemical activity, strength, and other novel characteristics [177]. The synthesis of green metal/metal oxide nanoparticles is less likely to produce environmentally hazardous byproducts. This is primarily due to the plant-derived mediated reducing, capping, and stabilizing agents. [178]. Currently, many researchers have inclined their interests toward the secondary metabolites from various parts of plants as a route of synthesis of metal/metal oxide nanoparticles [179]. Green metal/metal oxide nanoparticles are highly used in various applications such as antibacterial, antioxidant, anti-inflammatory, catalytic, and cytotoxic activities [180]. Even though few studies have been carried out on the green synthesis using aquatic and semiaquatic plant extracts, some earlier studies revealed that these plants are rich sources of stronger bioreductants for synthesizing metallic nanoparticles. Aquatic and semiaquatic plants mediated green synthesis of metallic nanoparticles showed a faster reaction process than other plants [181]. Mathur et al. described the synthesis of silver nanoparticles (AgNPs) using extracts of *Alternanthera sessilis* and *Withania somnifera* for their applications in the assays of cytotoxicity effects and antibacterial activities with promising results [182]. The phytochemicals from the stem, fruit, seeds, leaves, and flowers of *Alternanthera sessilis* have been used for the biosynthesis of gold nanoparticles (AuNPs) and AgNPs. These synthesized nanoparticles have antibacterial, antifungicidal, antiplasmodial, anti-inflammatory, anticancer, antidiabetic, antiviral, and antioxidant activities [183]. Other studies also displayed that AgNPs synthesized from extracts of *Alternanthera sessilis* demonstrated significant cytotoxicity effects on the breast cancer cells [184].

## 4. Conclusions and Future Prospectives

Aquatic and semiaquatic medicinal plant products have remarkable biological, pharmacological, agricultural, green materials synthesis, and industrial applications. They are also used as nutraceuticals, food, and medicine. These plants contain diverse natural compounds with numerous biological and chemical properties. Crude extracts or pure compounds from various parts of aquatic and semiaquatic plants possess potential nutritional and medicinal values. Phytochemicals are widely used to treat various infectious and noninfectious health ailments. Further, several aquatic and semiaquatic plants are used for the green synthesis of metal and metal oxide nanomaterials, which have shown many potential applications. Moreover, they are also helpful for various commercial product preparations. Even though these plant species have a wide range of phytochemicals with potential bioactive properties, enough research work is missing. Thus, this review article was designed. However, in the future, more extensive and specific research is required to investigate the natural phytochemicals from these aquatic and semiaquatic medicinal plants for various commercial uses.

## Figures and Tables

**Figure 1:** Some of the important aquatic medicinal plants. (a): *Acorus calamus*. (b): *Bacopa monnieri*. (c): *Centella asiatica*. (e): *Coix lacryma-jobi*. (f): *Enhydra fluctuans*. (d): *Centipeda minima*. (h): *Marsilea minuta*. (i): *Nelumbo nucifera*. (g): *Hedychium coronarium*. (j): *Nymphaea nouchali*. (l): *Rotula aquatic*. (k): *Persicaria hydropiper*. (n): *Pistia stratiotes*. (o): *Ammomum aromaticum*. (m): *Sphaeranthus indicus*. (r): *Sagittaria sagittifolia*. (p): *Hydrocotyle sibthorpioides*. (q): *Rumex maritimus.*

**Figure 2:** Some important semiaquatic medicinal plants. (a): *Ceratophyllum demersum*. (b): *Eleocharis dulcis*. (c): *Limnophila aromatica*. (e): *Marsilea minuta*. (d): *Ludwigia adscendens*. (f): *Nymphaea pubescens*. (g): *Rotala rotundifolia*. (h): *Ageratum conyzoides*. (i): *Ammannia baccifera*. (j): *Eclipta prostrate*. (l): *Hygrophila schulli*. (k): *Heliotropium indicum*. (m): *Spilanthes calva Candolle*. (n): *Vetiveria zizanoides.*

**Figure 3:** Chemical structures of some important phytochemical compounds obtained from various aquatic and semiaquatic plants: allantoin *α*-ionone *β*-asarone; avicularia *β*-cadinene catechin; hyperoside kaempferol linalool; querctrin rutin sabinene; triglyceride *α*-asarone *α*-terpinene; *β*-vetivone *β*-vetivene guaianolide; methoxy-cinnamaldehyde orientin 2*β*-hydroxyoleanolic acid; aromadendrene *β*-sitosterol apigenin-7-o-glucoside; *α*-humulene *β*-caryophyllene acacetin; luteolin 4′,7-dihydroxyflavone 1,8-cineole; baicalein-7-o-glucoside stigmasterol acorenone.

**Figure 4:** Phytochemical, biological, and some other applications of aquatic and semiaquatic medicinal plants.

**Table 1:** Some aquatic and semiaquatic medicinal plants with potential phytoconstituents and their applications.

Plant name	Family	Plant part used	Major phytochemicals	Type of extracts	Uses	References
*Aeschynomene aspera*	Fabaceae	Shoots	Glycosides, tannins, alkaloids, steroids, gums, and flavonoids	Crude extracts	(i) Treat cold, fever, and cough (ii) Increase semen consistency	[13]
*Ageratum conyzoides*	Asteraceae	Leaves and shoot	Rutin, quercitrin, avicularin, hyperoside, and catechin	Pure compounds	Used to treat fresh cuts and injuries and prepare traditional hair lotion	[14]
*Alternanthera philoxeroides*	Amaranthaceae	Shoot	*α*-Ionone and triglyceride	Pure compounds	Used to cure dysentery	[15]
*Ammannia auriculata*	Lythraceae	Leaf	Hydroxy-1-tetralone and *β*-sitosterol	Pure compounds	(i) Decrease fevers and rheumatic pains	[16]
*Caesulia axillaris*	Asteraceae	Whole plant part	4-Methyl-5-ergosta	Pure compound	Relieves cold, cough, dysentery, malaria, nasal congestion (ii) Healing wounds	[13, 17]
*Ceratophyllum demersum*	Ceratophyllaceae	Leaves	Apigenin-7-O-glucoside, benzyl acetate, and sesquiterpene	Pure compounds	(i) Relieves inflammatory effects, dysentery, epistaxis, fever, haematemesis, hemorrhoids, piles, hyperdipsia, intrinsic, scorpion sting, and ulcer (ii) Healing wounds	[18, 19]
*Coix aquatica*	Poaceae	Roots	Kaempferol and rutin	Pure compounds	Decrease the urination and menstrual complaints effects	[13]
*Cryptocoryne retrospiralis*	Araceae	Fresh tubers	Triterpene	Pure compound	Treats antiemetic, boils, burns, and vomiting during pregnancy	[20, 21]
*Cyperus haspan*	Cyperaceae	Rhizome	*α*-Ionone and triglyceride	Pure compounds	Treat fever and cough	[15, 22]
*Eleocharis dulcis*	Cyperaceae	Roots	Triglyceride and *β*-sitosterol	Pure compounds	Decreases abdominal pain, amenorrhea, cardiac risks, liver problems, nausea	[23]
*Fagopyrum esculentum*	Polygonaceae	Shoot	—	—	Used to treat the diabetic patient	[15, 24]
*Hygrophila auriculata*	Acanthaceae	Whole plant part	*β*-Cadinene	Pure compound	Decreases the anuria, blennorrhoea, catarrh, craw-craw, diuretic, hydropsy, menstruation, and stomach ache effects	[25, 26]
*Hygrophila polysperma*	Acanthaceae	Leaves and seeds	Terpinene-4-ol	Pure compound	Treat facial paralysis, hemiplegia, ear noise with headache, and stiff neck	[27]
*Lagenandra ovata*	Araceae	—	Sabinene and terpinen-4-ol	Pure compounds	(i) Relieves cardiac ailments (ii) Healing kidney disorders, skin problems, and swelling	[28]
*Limnophila aromatica*	Plantaginaceae	—	Hyperoside, quercitrin, avicularin, and catechin	Pure compounds	(i) Used as antimutagenic, mucus removal, antitumor, and pain killer (ii) Treats dysentery, elephantiasis, fever, indigestion, intestinal worms, and menstrual problems	[29]
*Limnophila indica*	Scrophulariaceae	Aerial parts	Triterpenoids and saponins	Crude extracts	Treats anthelmintic, antiseptic, dysentery, and elephantiasis	[13, 30]
*Lindernia Anagallis*	Scrophulariaceae	Whole plant	Acacetin and luteolin	Pure compounds	Treats asthma and gonorrhea	[13]
*Ludwigia adscendens*	Onagraceae	Whole plant	*α*-Terpineol	Pure compound	(i) Used as antimicrobial and anti-inflammatory (ii) Treats dysentery, skin diseases, and ulcers	[31, 32]
*Ludwigia octovalvis*	Onagraceae	Whole plant	Geraldone and acacetin	Pure compounds	Treats body ache, boil, diarrhea, fever, flatulence, heal dermatitis, toxemia, and ulcer	[33]
*Lysimachia nummularia*	Primulaceae	—	*β*-Asarone and *α*-asarone	Pure compounds	Treat cancer, stone lin syndrome, and wounds	[34]
*Marsilea minuta*	Marsileaceae	Leaves and root	Hyperoside, quercitrin, and avicularin	Pure compounds	Releaf biliousness, cough, headache, hypertension, insomnia, sleeping disorder, and spastic condition of leg muscles	[35]
*Monochoria hastata*	Pontederiaceae	Leaves	Rutin, protocatecheic acid, vanillic acid, and ferulic acid	Pure compounds	Used as anti-inflammatory agents	[36]
*Monochoria vaginalis*	Pontederiaceae	Leaves and flowers	*β*-Transocimenone, kaempferol, and solanin	Pure compounds	(i) Used as antioxidant, anti-inflammatory (ii) Treats asthma, coughs, stomach, toothache, swelling, and liver disorder	[37]
*Nymphaea pubescens*	Nymphaeaceae	Rhizome, roots	Orientin, *β*-D-glucopyranosyl	Pure compounds	Treats abortion, blood dysentery, dyspepsia, jaundice, leucorrhoea, menorrhagia, and piles disorders	[38]
*Nymphaea stellata*	Nymphaeaceae	Leaf	p-Cymene, *α*-selinene, and beta-gurjunene	Pure compounds	Treats stomach disorders	[39]
*Nymphoides hydrophylla*	Menyanthaceae	Leaves and seeds	Kaempferol and allantoin	Pure compounds	Treats eye diseases, fevers, insect bites, jaundice, scorpion sting, snakebite, and ulcer	[40]
*Nymphoides indica*	Menyanthaceae	Whole plant part	Kaempferol and allantoin	Pure compounds	Decreases fever, headache, rheumatism, and scabies disorders	[13]
*Polygonum barbatum*	Polygonaceae	Leaf, roots, and seeds	Kaempferol, baicalin, quercetin derivatives, and myricetin	Pure compounds	Treats bleeding from wounds, colic pain, cooling agent, and ulcers	[41]
*Rotala indica*	Lythraceae	Flower and leaves	*α*-Pinene and *β*-pinene	Pure compounds	Treats migraine, respiratory diseases, and stomach disorder	[33, 42]
*Rotala rotundifolia*	Lythraceae	Whole plant	Methoxycinnamaldehyde and *α*-terpinene	Pure compounds	(i) Used as antipyretic and antiswelling (ii) Treats cold, fever, cough, detoxication, diuresis, gonorrhea, menstrual cramps, piles, production in HepA2 cells, and suppression of HBV surface antigen (HBsAg)	[27, 43, 44]
*Vallisneria spiralis*	Hydrocharitaceae	Leaves	*β*-Vetispirene, vetiselinenol, husimol, *β*-vetinene, and *α*-vetivone	Pure compounds	(i) Treats leucorrhoea and stomachache	[45]

## Data Availability

No data were used to support this study.
